The article "Diagnosis of Heart Failure Complicated with Sleep Apnea Syndrome by Thoracic Computerized Tomography under Artificial Intelligence Algorithm" was published in 2022. Journal: Comput Math Methods Med.

# Diagnosis of Heart Failure Complicated with Sleep Apnea Syndrome by Thoracic Computerized Tomography under Artificial Intelligence Algorithm

**DOI:** 10.1155/2022/3795097

**Published:** 2022-05-09

**Authors:** Weihong Tian, Jinghua Li, Lan Ma

**Affiliations:** ^1^Department of Respiratory and Critical Care Medicine, Dingzhou People's Hospital, Dingzhou, 073000 Hebei, China; ^2^Department of Critical Care Medicine, Dingzhou People's Hospital, Dingzhou, 073000 Hebei, China; ^3^Department of Cardiology, Dingzhou People's Hospital, Dingzhou, 073000 Hebei, China

## Abstract

The aim of this study was to explore the application effect of thoracic computerized tomography (CT) under single threshold segmentation algorithm in the diagnosis of heart failure (HF) complicated with sleep apnea syndrome. 30 patients diagnosed with HF complicated with sleep apnea syndrome were chosen for the research. Another 30 patients without sleep apnea syndrome were selected as the control group, whose age, height, and weight were similar to those of the experimental group. Then, a model for thoracic CT image segmentation was proposed under the single threshold segmentation algorithm, and the faster region convolutional neural network (Faster RCNN) was applied to label the thoracic respiratory lesions. All the patients underwent thoracic CT examination, and the obtained images were processed using the algorithm model above. After that, the morphology of the patient's respiratory tract after treatment was observed. The results suggested that the improved single threshold segmentation algorithm was effective for the image segmentation of patient lesions, and the Faster RCNN could effectively finish the labeling of the lesion area in the CT image. The classification accuracy of the Faster RCNN was about 0.966, and the loss value was about 0.092. With CT scanning under the algorithm, it was found that the airway collapse of the posterior palatal area, retrolingual area, and laryngopharyngeal area of the sleep apnea syndrome patients was significantly greater than that of the control group (*P* < 0.05). But there was no significant difference of the collapse of the nasopharyngeal area between the two groups (*P* > 0.05). The single threshold segmentation algorithm had a better segmentation accuracy for thoracic CT images in patients with HF and sleep apnea syndrome, so it had a highly promising application prospect in the diagnosis of the disease.

## 1. Introduction

Obstructive sleep apnea (OSA) is a sleep-related breathing disorder that has a big impact on cardiovascular function. It is related to high blood pressure, coronary artery disease, arrhythmia, sudden cardiac death, and heart failure (HF), among which the HF affects about 23 million people in the world and about 5.8 million people in the United States, with a huge medical burden. In the United States, the incidence and prevalence rate of HF are increasing [1–3]. Mainly because of the aging of the population and the gradual extension of the HF patients' survival time through innovative therapies, the number of patients with HF is rising gradually. One of the factors for HF is just OSA. Compared with the ordinary population, the HF patients with reduced ejection fraction (HFrEF) or preserved ejection fraction (HFpEF) are more likely to have an onset of OSA. Therefore, there is some relationship between OSA and HF, and such a relationship has a great research significance pathophysiologically and clinically [4, 5]. Sleep apnea is characterized by partial or complete cessation of breathing during night sleep, leading to repeated awakening, oxygenated hemoglobin desaturation, and daytime sleepiness [6–8]. Apnea is defined as a complete stoppage of air flow for longer than 10 seconds or a hypopnea, which is the airflow partial cessation with 50% to 90% reduction in airflow for longer than 10 seconds, accompanied by a decrease in oxygen saturation (SaO_2_) by over 3% [9, 10]. According to the average prevalence rate, it is estimated that one in five adults has mild OSA, and one in fifteen adults has moderate OSA at least.

HF complicated with OSA is generally performed by computerized tomography (CT) examination. In recent years, artificial intelligence technology has been used in the segmentation of medical CT images, which greatly improves the segmentation effect of the lesion area [11]. The fully connected layer in the traditional convolutional neural network is optimized into a convolutional layer under the full convolutional neural network (FCNN), by which the complexity of the calculation is reduced and the segmentation efficiency is improved. Compared with the FCNN model, the single threshold segmentation algorithm can achieve a higher segmentation accuracy and is not limited by the input sample size [12, 13]. As the deep learning technology is applied for medical image processing and detection of lesions in images, the workload of manual processing can be reduced, and the issues such as poor diagnosis of subjective differences can be dealt with better.

Therefore, the model under deep learning was proposed in this research for the CT image analysis of OSA, and then, the diagnostic accuracy was compared with different diagnostic methods. Thus, a reference could be offered for improving the clinical diagnosis and treatment effects of patients with OSA.

## 2. Research Objects

Thirty patients who were diagnosed with sleep apnea syndrome in hospital were selected in the test group. They were monitored by night polysomnography (NPSG) and then were diagnosed. There were 24 males and 6 females in the group. They were 25-62 years old, with an average age of 45.54 ± 10.15 years old. Another 30 patients without sleep apnea syndrome were also selected as the control group, in which the age, height, and weight were similar to those of patients in the test group. All the patients have signed the informed consents, and all the researches have been approved by the ethics committee of the hospital.

Those who meet the diagnostic criteria for sleep apnea syndrome were included in the study, without craniofacial deformity, respiratory central diseases, and other malignant tumors. They agreed and accepted to be the participants in the study.

The exclusion criteria were described as follows. Those with incomplete imaging data, and who were unable to cooperate in the whole course of imaging examination, were out of the study.

## 3. Methodology

### 3.1. CT Examination

The whole-body low-dose CT examination was used. The scanning range was set from the top of the nasopharynx to below the glottis, the layer thickness was fixed as 5 mm, and the layer spacing was 2.5 mm. During the CT examination, all patients underwent the continuous upper airway scanning under four time phases, in the calm breathing, deep end inspiration, deep end expiration, and deep end inspiration with nose and mouth closed (Muller action). The patients lay supine with the head and neck stretched in the middle position. The raw image data was input to the workstation for postprocessing and measurement of various indexes. All the data were obtained by blind measurement. The thoracic CT scanning was also carried out. The image of upper airway was divided into 3 parts by the horizontalis of hard palate and the upper edge of epiglottis, including that of the nasopharyngeal area, oropharyngeal area, and laryngopharyngeal area. The nasopharyngeal area was from the nasopharyngeal dome to the horizontalis of hard palate, the oropharyngeal area was from the hard palate horizontalis to the upper edge of epiglottis, and the laryngopharyngeal area was from the upper edge of epiglottis to the upper edge of hyoid bone. Then, the oropharyngeal area was further divided into the posterior palatal area (the horizontalis of hard palate to the lower end of soft palate) and the retrolingual area (the lower end of soft palate to the upper edge of epiglottis). The images of upper airway were reconstructed in transverse, sagittal, and coronal planes, and the cross-sectional area of the nasopharynx, oropharynx, and laryngopharyngeal, the length and thickness of the soft palate were measured. From the above measured data, the airway collapse degree was calculated. In this study, the airway collapse degree = (end‐expiratory cross‐sectional area–end‐inspiratory cross‐sectional area)/end‐expiratory cross‐sectional area. At the same time, the internal surface of the airway was observed through a virtual endoscope.

### 3.2. CT Image Segmentation under Single Threshold Segmentation Algorithm

The single threshold segmentation algorithm was applied for the segmentation of the thoracic CT images. The following two main steps were included in this algorithm segmentation. Firstly, the threshold that needed to be segmented was determined and compared with the CT pixel value in the image; then, the pixels were divided. The calculation and selection of the segmentation threshold were the most important steps of the algorithm, and the iterative threshold method was used for it. The calculation steps of the iterative threshold were as follows.

Firstly, the maximum gray value and minimum gray value (*F*_max_ and *F*_min_) of the raw thoracic CT image were worked out, and the average gray range *k*_0_ was calculated via

(1) $$\begin{array}{c} k_{0}=\frac{F_{\max}+F_{\min}}{2}. \end{array}$$

Then, according to the average value *k*_0_, the gray average *D*_L_ and *D*_R_ of the foreground and background of the raw CT image were computed with

(2) $$\begin{array}{c} D_{\text{L}}=\frac{\sum_{F=0}^{K_{i}}H_{F}\cdot F}{\sum_{F=0}^{K_{i}}H_{F}}, \end{array}$$

(3) $$\begin{array}{c} D_{\text{R}}=\frac{\sum_{F=K_{i}+1}^{L-1}H_{F}\cdot F}{\sum_{F=K_{i}+1}^{L-1}H_{F}}. \end{array}$$

In the equations, *L* represented there were a total of *L* gray levels, *H*_*F*_ represented the number of pixels with a gray value of *F*, and *K*_*i*_ represented the threshold value in the *i*-th iteration.

When *K*_*i*+1_ = *K*_*i*_, at this time the iteration had a convergence to the stable threshold *k*_*i*_. At the moment, the iteration was ended, and the final threshold value *k*_*i*_ was taken as the segmentation threshold. Equation (4) was obtained at the same time.

(4) $$\begin{array}{c} k_{i}=\frac{D_{\text{L}}+D_{\text{R}}}{2}. \end{array}$$

However, it was found that, in the use the threshold segmentation algorithm, the raw CT image would be interfered by the peripheral background during segmentation, which resulted in a poor segmentation effect. Therefore, the erosion was utilized to erode the boundary area of the foreground pixels so that a more complete segmentation was achieved. The erosion is shown in Figure 1 in detail.

### 3.3. Thoracic CT Examination under Faster Region Convolutional Neural Network

For the intelligent detection of thoracic CT respiratory morphology with algorithms, faster region convolutional neural network (Faster RCNN) was introduced to detect the lesion area. The Faster RCNN mainly consisted of two parts, the region proposal network (RPN) and the region convolutional neural network (RCNN) [14]. The network classification model was used to extract the feature map, and then, the area of interest was generated and the pooling operation was carried out through the RPN. Each area of feature map of a specific size was extracted, and finally, the feature map was classified and given the probability value corresponding to the target category in the RCNN.

Then, the basic model of Visual Geometry Group (VGG) was applied for the extraction of the feature map. The convolution kernel sizes of some convolutional layers in the VGG model were 1 × 1 and 3 × 3, respectively. The activation function was a *softmax* function, and the *reshape* operation was carried out before and after the functional operation, so as to improve the classification effect.

The samples were input into the value model for training. The loss function of the model consisted of the RPN and the detector, but loss function was composed of a classification loss and a regression loss function. The mathematical expression was as

(5) $$\begin{array}{c} L\left(\left\{b_{i}\right\},\left\{d_{i}\right\}\right)=\frac{1}{N_{c}}\sum L_{c}\left(b_{i},b_{i}^{*}\right)+\alpha \frac{1}{N_{r}}\sum b_{i}^{*}L_{r}\left(d_{i},d_{i}^{*}\right). \end{array}$$

In Equation (5), *b*_*i*_ was the probability of the target region in the prediction box, while *b*^∗^_*i*_ was the multiclass label in *softmax* regression.

The mathematical expressions of classification loss *L*_c_ and regression loss *L*_r_ were expressed as

(6) $$\begin{array}{c} L_{\text{c}}\left(b_{i},b_{i}^{*}\right)=-\log\left(b_{i}^{*}b_{i}+\left(1-b_{i}^{*}\right)\left(1-b_{i}\right)\right), \end{array}$$

(7) $$\begin{array}{c} L_{\text{r}}\left(d_{i},d_{i}^{*}\right)=R\left(d_{i}-d_{i}^{*}\right). \end{array}$$

In the above two equations, *R* represented the smooth *L*1 function, and *d*_*i*_ was the offset of the prediction box during RPN training; *d*_*i*_^∗^ and *d*_*i*_ had the same dimension.

With the iteration of the loss function, the parameters of the *softmax* classifier were further optimized and clarified, which made it gain a discriminative function for different training samples.

### 3.4. Statistical Processing

SPSS 19.0 was used for the statistical analysis. Measurement data conforming to normal distribution were expressed as the average ± standard deviation, and comparisons between groups were analyzed by independent sample *t*-test. Measurement data that did not conform to normal distribution were expressed by the median value and four-point position representation, and nonparametric rank sum test was used to analyze the differences between groups. Enumeration data was measured by *n*(%), and the comparison of differences between groups was analyzed by chi-square test. *P* < 0.05 showed the difference was statistically significant.

## 4. Results

### 4.1. Segmentation Performance Analysis of Single Threshold Segmentation Algorithm

With the single threshold segmentation algorithm of artificial intelligence, the selected thoracic CT undersampled images were segmented and optimized, and then, the preprocessed thoracic CT images were obtained. The comparison result is shown in Figure 2, as the area inside the box was the range of feature extraction, and the dotted line indicated the feature contour extracted by this algorithm. It could be observed from Figure 2 that, in the unprocessed original thoracic CT images, the interference of irrelevant regions was more obvious, and some structures were blurred. After being processed by a single threshold segmentation algorithm, the CT images with clearer structure were output. In this way, the quality of image segmentation was improved, the amount of subsequent calculations was reduced, and the foundation was formed for the subsequent further segmentation of specific tissues.

### 4.2. Verification of the Faster RCNN Model

As the Faster RCNN model was trained, it was shown that when the number of training iterations reached 10, the classification accuracy and loss value of the model had been gradually stabilized. The classification accuracy of the Faster RCNN model was about 0.966, and the loss value was about 0.092.

As shown in Figure 3, the trained Faster RCNN was effective to detect the respiratory tract morphology in thoracic CT images. The marked area in Figure 3 was just the lesion location was labeled under the Faster RCNN.

### 4.3. General Data of the Patients

The baseline information of the patients in the test group and the control group is shown in Table 1. It can be known that the differences between that of patients in two groups were not statistically significant (*P* > 0.05), in the age, weight, gender, and height. Therefore, the results are comparable.

### 4.4. Comparison of Cardiopulmonary Function Indexes between Two Groups

The cardiopulmonary function of the patients in the test group and the control group was measured; the indexes measured were compared then. As shown in Figures 4 and 5, the left ventricular end-systolic dimension (LVESD) and left ventricular end-diastolic dimension (LVEDD) of the control group were significantly lower than those of the test group (*P* < 0.05).

### 4.5. Comparison of Imaging Results between the Two Groups

The patients in the two groups underwent the CT scanning of their upper airway. It is shown in Figure 6 that the airway collapse of the posterior palatal area, retrolingual area, and laryngopharyngeal area of the sleep apnea syndrome patients was significantly greater than that in the control group (*P* < 0.01). However, there was no significant difference in the collapse of the nasopharynx between the two groups (*P* > 0.05).

## 5. Discussion

OSA is characterized by repeated pharynx collapse during sleep. Patients usually have a narrow, highly compliant pharynx. It easily collapses during sleep when the pharyngeal dilator muscles contract normally, which results in airway narrowing (hypopnea) or obstruction (apnea). Many patients are obese, and fat deposits around the pharynx may be a part of the causes of the narrowing of the pharynx [15]. Relevant evidence shows that the lateral displacement of fluid that accumulates in the legs during the day can lead to edema of the peripharyngeal structure during sleep, which makes the patient very susceptible to OSA.

The mechanical, chemical, neurohumoral, and inflammatory mechanisms caused by OSA are usually harmful to the cardiovascular system. During the onset of mechanical airflow obstruction, attempting to inhale would directly cause excessive drop, hypoxia, and arousal of intrathoracic pressure. A drop of intrathoracic pressure will increase the transmural pressure of the left ventricle, thereby the load is increased. Such a pressure drop will also lead to increased venous return, the right ventricle dilatation as the ventricular septum shift to the left, and a decreased left ventricular filling. The decreased left ventricular filling and increased afterload will cause a decrease of stroke volume at last. Hypoxia, sleep arousal, and significantly repeated increases in systemic blood pressure due to sympathetic nervous activity (SNA) are also brought by OSA [16, 17]. SNA would get a further development by reducing the stroke volume, inhibiting the sympathetic inhibitory effect of lung extension receptors through apnea, or both. When the SNA is strengthened, the increased left ventricular afterload together with increased heart rate will lead to a mismatch between myocardial oxygen supply and demand, which makes patients acutely susceptible to myocardial ischemia and arrhythmia and chronically susceptible to left ventricular hypertrophy, left ventricular enlargement, and HF [18, 19].

For the diagnosis of HF complicated with sleep apnea syndrome, the common clinical method is CT, which has the characteristics like it can be operated simply, economical, and practical. It has a good presentation effect on thoracic diseased tissues and can meet the needs of clinical diagnosis of HF combined with sleep apnea syndrome in general. However, if to improve the efficiency and accuracy of clinical diagnosis further, the resolution of CT images is still a little low, which may cause some details of diseases be ignored. Therefore, it is necessary to improve the quality of CT images. In recent years, the use of artificial intelligence algorithms for processing medical images is a major trend in medical imaging [20]. Threshold segmentation on the basis of intelligent algorithms is the most common method for image segmentation. In a grayscale image under the algorithm in this work, the pixel value in the target area was similar to the adjacent pixel value in the background, and the pixel values of different target areas are different. The region segmentation was then processed according to the peak value of the target region displayed on the histogram [21, 22]. For traditional segmentation algorithms are affected by image noise and other factors, the poor segmentation is produced. The single threshold segmentation model has had an excellent achievement in the segmentation of medical images [23, 24].

In this research, the single threshold segmentation algorithm-based CT technology was applied for diagnosing HF complicated with sleep apnea syndrome. The results suggested that the image quality processed by the single threshold segmentation algorithm was better notably, and the distinctions between lesions and tissues were also highly improved. The single threshold algorithm showed a better segmentation performance compared with the traditional algorithm. In the diagnosis with CT technology under single threshold segmentation algorithm, remarkable differences were shown between the patients and the normal people of the control group. This illustrated that the single threshold segmentation algorithm-based CT technology had a grander application prospect and value in the diagnosis of HF complicated with sleep apnea syndrome.

## 6. Conclusion

With deep learning technology, the thoracic CT image segmentation and classification were done for the improvement of clinical diagnosis of patients with HF complicated with sleep apnea syndrome. CT technology under the singular threshold segmentation algorithm could segment the lesions well and accurately of HF complicated with sleep apnea syndrome patients. Under the diagnosis with this technology, the imaging characteristics were presented with obvious differences between the patients and normal control population. It was proved that single threshold segmentation algorithm-based CT technology possessed a greater application value as well as prospect in the diagnosis of HF complicated with sleep apnea syndrome.

However, there were still some limitations in this study. Deep learning was applied and studied only for the segmentation and classification of the lesion areas in the patients' CT image; its application for the evaluation of the patients' CT image after treatment was not included. Meanwhile, only one imaging diagnosis method was analyzed, and more imaging diagnosis methods and in-depth evaluation of the impact of different indexes on the prognosis of patients needed further researches. In conclusion, the results of this study can offer an effective improvement to the diagnosis of patients with HF and sleep apnea syndrome, guidance for subsequent clinical treatment, and theoretical basis for follow-up researches of imaging examination methods.

## Figures and Tables

**Figure 1:** Diagram of corrosion operation. A represented any point in the shaded part, while B stood for the structural element.

**Figure 2:** Comparison of the segmentation effect of single threshold segmentation algorithm on thoracic CT images. The area inside the red box was the feature extraction range; the dotted line was the feature contour extracted by the algorithm.

**Figure 3:** Label of respiratory tract morphological lesions under the Faster RCNN.

**Figure 4:** Comparison of the cardiac function indexes between two groups. ∗ indicated that the difference between groups was statistically significant, *P* < 0.05.

**Figure 5:** Comparison of the pulmonary function indexes between two groups. FEV1: forced expiratory volume in one second; FVC: forced vital capacity. ∗ indicated the statistically significant difference between groups, *P* < 0.05.

**Figure 6:** Comparison of imaging results between the two groups. ∗ indicated that the differences between groups were of statistical significance, *P* < 0.05.

**Table 1:** Comparison of patients' baseline information between the two groups.

Items		Test group (*n* = 30)	Control group (*n* = 30)	Statistic value	*P*
Age (years old)		45.54 ± 10.15	47.69 ± 11.12	*t* = 0.771	0.441
Height (m)		1.66 ± 0.08	1.65 ± 0.10	*t* = 0.453	0.652
Weight (kg)		67.52 ± 10.51	66.85 ± 11.86	*t* = 0.317	0.752
Gender (*n*/%)	Males	24	22	*χ* ^2^ = 0.839	0.334
	Females	6	8		

## Data Availability

The data used to support the findings of this study are available from the corresponding author upon request.

## References

[1] Borel A. L. (2019). Sleep apnea and sleep habits: relationships with metabolic syndrome. *Nutrients*.

[2] Gulotta G., Iannella G., Vicini C. (2019). Risk factors for obstructive sleep apnea syndrome in children: state of the art. *International Journal of Environmental Research and Public Health*.

[3] Javaheri S., Barbe F., Campos-Rodriguez F. (2017). Sleep apnea: types, mechanisms, and clinical cardiovascular consequences. *Journal of the American College of Cardiology*.

[4] Dempsey J. A. (2019). Central sleep apnea: misunderstood and mistreated!. *F1000Research*.

[5] Drager L. F., McEvoy R. D., Barbe F., Lorenzi-Filho G., Redline S., INCOSACT Initiative (International Collaboration of Sleep Apnea Cardiovascular Trialists) (2017). Sleep apnea and cardiovascular disease: lessons from recent trials and need for team science. *Circulation*.

[6] Arnaud C., Bochaton T., Pépin J. L., Belaidi E. (2020). Obstructive sleep apnoea and cardiovascular consequences: pathophysiological mechanisms. *Archives of Cardiovascular Diseases*.

[7] Mencar C., Gallo C., Mantero M. (2020). Application of machine learning to predict obstructive sleep apnea syndrome severity. *Health Informatics Journal*.

[8] Santos A., Walsh H., Anssari N., Ferreira I., Tartaglia M. C. (2020). Post-concussion syndrome and sleep apnea: a retrospective study. *Journal of Clinical Medicine*.

[9] Otto-Yáñez M., Torres-Castro R., Nieto-Pino J., Mayos M. (2018). Síndrome de apneas-hipopneas obstructivas del sueño y accidente cerebrovascular [Obstructive sleep apnea-hypopnea and stroke]. *Medicina (B Aires)*.

[10] McDermott M., Brown D. L., Chervin R. D. (2018). Sleep disorders and the risk of stroke. *Expert review of neurotherapeutics*.

[11] Sahiner B., Pezeshk A., Hadjiiski L. M. (2019). Deep learning in medical imaging and radiation therapy. *Medical Physics*.

[12] Huang Y., Hu G., Ji C., Xiong H. (2020). Glass-cutting medical images via a mechanical image segmentation method based on crack propagation. *Nature Communications*.

[13] Shang H., Zhao S., Du H., Zhang J., Xing W., Shen H. (2020). A new solution model for cardiac medical image segmentation. *Journal of Thoracic Disease*.

[14] Teng L., Li H., Karim S. (2019). DMCNN: a deep multiscale convolutional neural network model for medical image segmentation. *Journal of Healthcare Engineering*.

[15] Sun C., Xu Y., Luo C., Li Q. (2020). Relationship between enuresis and obstructive sleep apnea-hypopnea syndrome in children. *The Journal of International Medical Research*.

[16] Masa J. F., Pépin J. L., Borel J. C., Mokhlesi B., Murphy P. B., Sánchez-Quiroga M. Á. (2019). Obesity hypoventilation syndrome. *European Respiratory Review*.

[17] Oliveira L. M., Nitrini R., Román G. C. (2019). Normal-pressure hydrocephalus: a critical review. *Dementia & Neuropsychologia*.

[18] Kimura H., Ota H., Kimura Y., Takasawa S. (2019). Effects of intermittent hypoxia on pulmonary vascular and systemic diseases. *International Journal of Environmental Research and Public Health*.

[19] Liang J., Zhang X., Luo Y., Wang T., Sun L., Huang S. (2018). The impact of respiratory events on the autonomic nervous system during sleep. *International Heart Journal*.

[20] Wang J. Z., Shi X. J., Yao X. C., Ren J., Du X. R. (2021). Deep learning-based CT imaging in diagnosing myeloma and its prognosis evaluation. *Journal of Healthcare Engineering*.

[21] Xie D. H., Lu M., Xie Y. F., Liu D., Li X. (2019). A fast threshold segmentation method for froth image base on the pixel distribution characteristic. *PLoS One*.

[22] Friedli L., Kloukos D., Kanavakis G., Halazonetis D., Gkantidis N. (2020). The effect of threshold level on bone segmentation of cranial base structures from CT and CBCT images. *Scientific Reports*.

[23] Zheng W., Wang Q., Wang Y., Guo F., Wang X., Yu T. (2017). Threshold segmentation of pulmonary subsolid nodules on CT images: detection and quantification of the solid component. *Zhongguo Fei Ai Za Zhi*.

[24] Pfaehler E., Burggraaff C., Kramer G. (2020). PET segmentation of bulky tumors: strategies and workflows to improve inter-observer variability. *PLoS One*.

